RETRACTED

# Long Non-coding RNA H19 Deteriorates Hypoxic-Ischemic Brain Damage by Interacting with MicroRNA-140-5p and STAT3

**DOI:** 10.1186/s11671-022-03666-8

**Published:** 2022-04-05

**Authors:** Qian Lu, Hai Man Hou, Shuo Li, Jing Yuan, Han Liu, Yuming Xu

**Affiliations:** Department of Neurology, The First Affiliated Hospital of Zhengzhou University, 1 Jianshe East Road, Erqi District, Zhengzhou, 450000 Henan China

**Keywords:** Hypoxic-ischemic brain damage, Long non-coding RNA H19, MicroRNA-140-5p, Signal transducer and activator of transcription 3, Oxygen glucose deprivation, Angiogenesis, Apoptosis, Migration

## Abstract

**Objective:**

Even though extensive studies have surveyed long non-coding RNA (lncRNA)-related networks in hypoxic-ischemic brain damage (HIBD), the concrete function of lncRNA H19 (H19) in HIBD is still in ambiguity. Therein, this work intends to decipher H19-related network of microRNA (miR)-140-5p and signal transducer and activator of transcription 3 (STAT3) in HIBD.

**Methods:**

Brain microvascular endothelial cells (BMECs) from BALB/c mice were isolated and induced by oxygen glucose deprivation (OGD). OGD-induced BMECs were transfected with depleted or restored H19, miR-140-5p or STAT3, and cell apoptosis, migration and angiogenesis were examined. H19, miR-140-5p and STAT3 expression and their internal connections were tested.

**Results:**

H19 and STAT3 were overexpressed while miR-140-5p was down-regulated in OGD-induced BMECs. H19 or STAT3 knockdown, or miR-140-5p restoration repressed apoptosis and improved migration and angiogenesis of OGD-induced BMECs. MiR-140-5p restoration negated the impacts of up-regulated H19 on OGD-induced BMECs. H19 bound to miR-140-5p to modulate STAT3 expression.

**Conclusion:**

The work illustrates that depleting H19 or STAT3 or restoring miR-140-5p attenuates HIBD and supplies a novel perspective for HIBD management.

**Supplementary Information:**

The online version contains supplementary material available at 10.1186/s11671-022-03666-8.

## Introduction

Hypoxic-ischemic brain damage (HIBD) is a predominant contributor to morbidity and mortality in preterm and term newborns [1]. It is reported that 7 out of every 1000 preterm infants and 3 out of every 1000 term infants are diagnosed with HIBD. Of these, only about 60% survive the neonatal period, and about 30% further suffer from long-term neurological diseases, such as learning defects and visual impairment [2]. The available approaches for HIBD management consist of neuroprotective agents, ibuprofen, stem cell therapy and hypothermia therapy [3]. At present, the task to delve out potential targeted therapy is put on the agenda.

RETRACTED

The therapeutic efficacy of long non-coding RNAs (lncRNAs) in HIBD has been previously explored. For instance, depletion of lncRNA metastasis-associated lung adenocarcinoma transcription 1 could protect hippocampal neurons against HIBD by interacting with microRNA (miR)-429 [4] and lncRNA growth arrest-specific transcript 5 down-regulation promotes neurological function recovery and reduces brain infarction in rats with HIBD [5]. In terms of the functional role of lncRNA H19 (H19), there is a research explaining that H19 mediates cell apoptosis and cerebral damage in hypoxic ischemia encephalopathy (HIE) [6]. Lately, an investigation has summarized that H19 protects neurons and regulates oxidative stress injury induced by ischemia/reperfusion (I/R) [7]. miR-140-5p is a mediator of angiogenesis in ischemic stroke (IS) [8], and it can relive neuroinflammation and ameliorate intracerebral hemorrhage (ICH)-induced brain injury [9]. Precisely, miR-140-5p can improve neuronal survival in rats with HIBD [10]. Signal transducer and activator of transcription 3 (STAT3) is a crucial actor in cell proliferation, angiogenesis and survival of tissues [10, 11]. Studies have elucidated that STAT3 signaling inhibition attenuates blood–brain barrier abnormality in oxygen glucose deprivation/reoxygenation (OGD/R)-treated cells [12], and depleted STAT3 protects brain microvascular endothelial cells (BMECs) which are injured by OGD and hemin in advance [13]. Interestingly, H19 has been indicated to sponge miR-140 [14]. Taken together, the integrated function of these three factors is not comprehended clearly. Thereafter, this study was launched to elaborate their combined interplay in HIBD.

## Materials and Methods

### Ethics Statement

All experiments were approved and supervised by the ethics committee of The First Affiliated Hospital of Zhengzhou University. The animal experiment plan was approved by the Animal Ethics Committee of The First Affiliated Hospital of Zhengzhou University.

### Materials

Materials used in our study are listed in Additional file 1: Table S1.

### Isolation and Identification of BMECs

BALB/c mice (Laboratory Animal Center of Zhengzhou University, Zhengzhou, China), male and female were 4–6 weeks old and weighed 15–20 g. The mice were euthanized by cervical vertebra dislocation. The mouse whole brain and separated cerebral cortex were placed in high-glucose Dulbecco’s modified eagle medium (DMEM), shed into 1 mm^3^ and incubated with 0.1% type II collagenase (containing 20 μmol/L DNase I) in water bath. After centrifugation, the samples were added with 20% bovine serum albumin and centrifuged once again to remove nerve tissues and blood vessels. Afterwards, the brain tissues were detached by 0.1% trypsin, centrifuged, supplemented with 20% newborn calf serum and centrifuged once again. The white-yellow layer was the purified microvascular segment. The microvascular segment was added with DMEM, centrifuged and appended by a complete medium (20% fetal bovine serum (FBS), endothelial growth factor, 1 g/L heparin sodium, 1 × 10^5^ U/L penicillin, 100 mg/L streptomycin, and 2 mmol/L L-glutamine). The cell suspension was seeded, with the medium changed 12–24 h later and then once every day. Cultured for 7–9 days, the cells were adhered to the wall and detached with 0.25% trypsin. Only the cells detached in the first 5 min were utilized for cell experiments. BMECs were identified by immunofluorescence staining of endothelial cell specific marker CD31, and cell staining was observed under a fluorescent microscope. The morphology of BMECs was observed under an inverted phase contrast microscope [15].

RETRACTED

### OGD Modeling and Transfection of BMECs

BMECs was induced by OGD to stimulate HIBD in vitro [16]. BMECs of passage 3–4 were trypsinized and seeded on a culture plate with 5 × 10^4^ cells/well. Upon complete confluence, BMECs were cultured in glucose-free Hanks solution and incubated under OGD (95% N_2_ and 5% O_2_) for 0, 2, 4, 6 and 8 h, respectively. Then, BMECs were transferred into a medium containing 10% FBS and incubated under normal oxygen conditions (37 °C, 5% CO_2_).

BMECs were respectively transfected with H19 interference negative control (sh-NC); H19 interference plasmid (sh-H19); overexpression of empty vector (oe-NC); H19 overexpression plasmid (oe-H19); mimic NC; miR-140-5p mimic; inhibitor NC; miR-140-5p inhibitor; sh-H19 and inhibitor NC; sh-H19 and miR-140-5p inhibitor; STAT3 interference plasmid (sh-NC); STAT3 interference plasmid (sh-STAT3); STAT3 overexpression plasmid (oe-STAT3); STAT3 overexpression plasmid NC (oe-NC). The above oligonucleotides and plasmids were designed and synthesized by GenePharma (Shanghai, China). Transfection was performed in line with the instructions of Lipofectamine 2000 reagent (Invitrogen, CA, USA). At 24 h post transfection, BMECs were processed with OGD for 6 h.

### 3-(4,5-Dimethylthiazol-2-yl)-2,5-Diphenyltetrazolium Bromide (MTT) Assay

BMECs suspension (200 μL) was seeded in 96-well plates at 1 × 10^4^ cells/well and cultured to complete confluence. After transfection and OGD induction, BMECs were incubated with MTT solution (5 g/L, 20 μL) for 1 h and with 150 μL dimethyl sulfoxide for 5 min. Absorbance (490 nm) values were recorded on a microplate reader.

### Flow Cytometry

Annexin V-fluorescein isothiocyanate (FITC) Apoptosis Detection Kit was utilized to detect apoptosis rate. BMECs (5 × 10^3^) were resuspended in 500 μL binding buffer and reacted with 5 μL Annexin V-FITC and 5 μL PI solution for 15 min. a flow cytometer (BD Biosciences, Franklin Lakes, NJ, USA) was employed for examining cell apoptosis rate.

RETRACTED

### Transwell Assay

Migration ability of BMECs was tested by Transwell assay. BMECs (1 × 10^5^) were placed in the upper side of Transwell chamber (BD Bioscience) filled with serum-free medium (100 μL), and the lower chamber was filled with 10% FBS (600 μL). Incubated for 24 h, BMECs on the matrigel were swiped away while those migrated were pre-fixed by 95% ethanol, stained with 1% crystal violet solution and counted under an inverted microscope in 5 randomly-selected fields.

### Angiogenesis Detection

Angiogenesis was tested in compliance with the instructions of the angiogenesis detection kit (Millipore, MA, USA). The pre-thawed Matrigel (BD Biosciences) was placed in the 96-well plate for polymerization. BMECs were seeded on the Matrigel at 1 × 10^4^ cells/well and hatched for 12 h. BMECs were observed under an inverted microscope in 5 fields and the number of formed tubes in each field was counted and averaged.

### Dual Luciferase Reporter Gene Assay

H19 or STAT3 3’untranslated region (UTR) containing the miR-140-5p target site were cloned into the pMIR-Report Luciferase vector (Ambion, Austin, TX, USA) downstream of the firefly luciferase gene to produce pmiR-RB-H19-wild type (WT) or pmiR-RB-STAT3 3′UTR-WT. Then, the binding site containing miR-140-5p was mutated to form pmiR-RB-H19-mutant type (MUT) or pmiR-RB-STAT3 3′UTR-MUT. BMECs were cotransfected with reporter plasmids and miR-140-5p mimic or its NC with Lipofectamine 2000. Firefly luciferase activities were measured using the Dual Luciferase Assay (Promega, Madison, WI) 48 h after transfection and the results were normalized with Renilla luciferase.

### RNA Pull-Down Assay

Three biotinylated miRNA sequences were designed and synthesized: Bio-miR-140-5p-WT, Bio-miR-140-5p-MUT, and Bio-NC. BMECs with 80–90% confluence were transfected with the three miRNA sequences, respectively. At 48 h post transfection, BMECs were lysed and the lysate was incubated with M-280 streptavidin-coated magnetic beads (Sigma-Aldrich, CA, USA). The magnetic beads were washed and protein-nucleic acid complex adsorbed by the magnetic beads was eluted and lysed by Trizol to extract RNA. Reverse transcription quantitative polymerase chain reaction (RT-qPCR) was utilized to test H19 expression.

### RT-qPCR

In line with the instructions of Trizol reagent (Life Tech, CA, USA), total RNA was extracted from BMECs. RNA concentration and quality were tested by an ultraviolet spectrophotometer. RT-qPCR was carried out on a 7500 Real-time PCR system (Applied Biosystems, CA, USA). For LncRNA and mRNA analysis, cDNA was synthesized using the TaKaRa PrimeScript RT reagent kit (TaKaRa, Dalian, China). Quantitative PCR was conducted using TaKaRa SYGB Premix EX Taq (Tli RNaseH Plus, CA). For miRNA analysis, the One Step PrimeScript miRNA cDNA Synthesis Kit (TaKaRa) and the SYBR PrimeScriptTM miRNA RT-PCR Kit (TaKaRa) were used.  Glyceraldehyde-3-phosphate dehydrogenase (GAPDH) was an internal control for H19 and STAT3 while U6 was that for miR-140-5p. The primer sequences were demonstrated in Additional file 1: Table S2. The relative expression level was calculated by 2^−ΔΔCt^ method.

RETRACTED

### Western Blot Assay

BMECs were washed with PBS and then harvested using ice-cold RIPA lysis buffer containing protease inhibitor and protein phosphotase inhibitor. Protein concentration of total cell lysate was measured using BCA reagent (Pierce, Rockford, IL). Separated by 10% sodium dodecyl sulphate polyacrylamide gel electrophoresis, the protein was transferred to a polyvinylidene fluoride membrane and blocked. After that, the protein membrane was probed with the corresponding primary antibodies STAT3 (1:1000, Cell Signaling Technologies, MA, USA) and GAPDH (1:2500) overnight, and with the horseradish peroxidase-labeled secondary antibody (1:5000, both from Abcam, MA, USA). The developed membrane was photographed by an imager.

### RNA-Binding Protein Immunoprecipitation (RIP) Assay

Magna RIP RNA-Binding Protein Immunoprecipitation Kit (Millipore) was applied to RIP assay. BMECs were lysed by human anti-Ago2 (Abcam) or immunoglobulin G (IgG)-conjugated magnetic beads (Abcam) in RIP lysis buffer, and incubated with proteinase K and Rnase inhibitor to isolate immunoprecipitated RNA. The purified RNA was assessed by RT-qPCR to confirm the existence of binding site between H19 and miR-140-5p.

### Statistical Analysis

Data were statistically analyzed by SPSS21.0 (SPSS, Inc, Chicago, IL, USA) and GraphPad Prism 6.0 (GraphPad Software Inc.). The data were expressed as mean ± standard deviation. Discrepancy between two groups was evaluated by t test and that among multiple groups by one-way analysis of variance (ANOVA), followed by Tukey’s post hoc test. *P* < 0.05 stood for statistical significance.

## Results

### Identification and Morphological Observation of BMECs

Immunofluorescence staining was applied to detect CD31 and the results manifested that CD31-positive cells (green fluorescence) accounted for more than 90% of all cells (Fig. 1A). Under the light microscope, BMECs were long fusiform, with slightly stained nuclei and obvious cell membrane; BMECs were arranged irregularly (Fig. 1B).

RETRACTED

**Fig. 1:** Identification and morphological observation of BMECs; H19 and STAT3 are overexpressed while miR-140-5p is down-regulated in OGD-induced BMECs. **A** CD31-positive cells detected by immunofluorescence staining; **B** Observation of morphology of BMECs; **C** Cell viability after OGD treatment detected by MTT assay; **D**, **E** H19, miR-140-5p and STAT3 expression at 0, 2, 4, 6, and 8 h of OGD treatment detected by RT-qPCR and western blot assay; N = 3. The data were expressed as the mean ± standard deviation

### H19 and STAT3 are Overexpressed While miR-140-5p is Down-Regulated in OGD-Induced BMECs

For identifying the role of H19 in BMECs during HIBD, BMECs were induced by OGD to establish in vitro cell models. BMECs viability was measured at 0, 2, 4, 6, 8 h after OGD treatment (Fig. 1C). It was manifested that OGD reduced BMECs viability in a time-dependent manner (*P* < 0.05). H19, miR-140-5p and STAT3 expression in BMECs was tested and the findings suggested that OGD-treated BMECs showed increased H19 and STAT3 expression and decreased miR-140-5p expression (Fig. 1D, E). It is suggested that lncRNA H19 /miR-140-5p/STAT3 axis might play important roles in BMECs response to OGD treatment.

### H19 Knockdown Represses Apoptosis and Improves Migration and Angiogenesis of OGD-Induced BMECs

sh-H19 or oe-H19 was transfected into BMECs. RT-qPCR revealed that (Fig. 2A) sh-H19 decreased H19 expression while oe-H19 elevated H19 expression. In terms of cell viability and apoptosis, restored H19 impaired cell viability, enhanced cell apoptosis rate. Silenced H19 functioned in an opposite way to restored H19 (Fig. 2B, C).

**Fig. 2:** H19 knockdown represses apoptosis and improves migration and angiogenesis of OGD-induced BMECs. **A** H19 expression in sh-H19- or oe-H19-transfected and OGD-induced BMECs detected by RT-qPCR; **B** Viability of sh-H19- or oe-H19-transfected and OGD-induced BMECs detected by MTT assay; **C** Apoptosis of sh-H19- or oe-H19-transfected and OGD-induced BMECs detected by flow cytometry; **D** Cell migration of sh-H19- or oe-H19-transfected and OGD-induced BMECs detected by Transwell assay; **E** Angiogenesis of sh-H19- or oe-H19-transfected and OGD-induced BMECs detected by Matrigel method; N = 3; *P < 0.05 compared with the oe-NC group; ^#^*P* < 0.05 compared with the si-NC group. The data were expressed as the mean ± standard deviation

OGD treatment suppressed migration and angiogenesis of BMECs. Moreover, H19 up-regulation obstructed OGD-induced BMECs to migrate and form tubes. On the contrary, H19 down-regulation reinforced migration and angiogenesis of OGD-induced BMECs (Fig. 2D, E).

RETRACTED

### MiR-140-5p Restoration Represses Apoptosis and Improves Migration and Angiogenesis of OGD-Induced BMECs

Owing to that miR-140-5p expression in OGD-treated BMECs differed from that in normal BMECs, gain- and loss-of-function assay was carried out in BMECs. RT-qPCR displayed that miR-140-5p mimic elevated miR-140-5p expression while miR-140-5p inhibitor suppressed miR-140-5p expression in OGD-induced BMECs (Fig. 3A). Moreover, miR-140-5p suppression destroyed cell viability, and migration and angiogenesis, and heightened apoptosis rate. However, miR-140-5p enhancement caused complete opposite effects on these parameters in OGD-treated BMECs (Fig. 3B–E).

**Fig. 3:** miR-140-5p restoration represses apoptosis and improves migration and angiogenesis of OGD-induced BMECs. **A** miR-140-5p expression in miR-140-5p inhibitor- or miR-140-5p mimic-transfected and OGD-induced BMECs detected by RT-qPCR; **B** Viability of miR-140-5p inhibitor- or miR-140-5p mimic-transfected and OGD-induced BMECs detected by MTT assay; **C** Cell apoptosis of miR-140-5p inhibitor- or miR-140-5p mimic-transfected and OGD-induced BMECs detected by flow cytometry; **D** Cell migration ability of miR-140-5p inhibitor- or miR-140-5p mimic-transfected and OGD-induced BMECs detected by Transwell assay; **E** Angiogenesis of miR-140-5p inhibitor- or miR-140-5p mimic-transfected and OGD-induced BMECs detected by Matrigel method; N = 3; *P < 0.05 compared with the inhibitor NC group; ^#^*P* < 0.05 compared with the mimic NC group. The data were expressed as mean ± standard deviation

### MiR-140-5p Restoration Negates the Impacts of Up-Regulated H19 on OGD/R-Induced BMECs

The bioinformatics website Starbase (http://starbase.sysu.edu.cn/) predicted the binding site of H19 and miR-140-5p (Fig. 4A). Dual luciferase reporter gene assay revealed that miR-140-5p up-regulation impaired luciferase activity of the reporter vector containing H19-WT but had no effects on the luciferase activity of the reporter vector containing H19-MUT (Fig. 4B). Further detected by RNA pull-down assay, it was indicated that H19 expression was elevated by Bio-miR-140-5p-WT but not Bio-miR-140-5p-MUT (Fig. 4C). RIP assay results outlined that the enrichment of H19 and miR-140-5p was enhanced under anti-Ago2 (Fig. 4D).

**Fig. 4:** miR-140-5p restoration negates the impacts of up-regulated H19 on OGD-induced BMECs. **A** The binding site of H19 and miR-140-5p detected by bioinformatics website; **B** The binding relationship verified by dual luciferase report gene assay; **C** The binding relationship between H19 and miR-140-5p detected by RNA pull-down assay; **D** The enrichment level of H19 and miR-140-5p detected by RIP assay; **E**, **F** miR-140-5p expression in oe-H19- and miR-140-5p-mimic-transfected and OGD-induced BMECs detected by RT-qPCR; **G** Viability of oe-H19- and miR-140-5p-mimic-transfected and OGD-induced BMECs detected by MTT assay; **H** Cell apoptosis of oe-H19- and miR-140-5p-mimic-transfected and OGD-induced BMECs detected by flow cytometry; **I** Cell migration of oe-H19- and miR-140-5p-mimic-transfected and OGD-induced BMECs detected by Transwell assay; **J** Angiogenesis of oe-H19- and miR-140-5p-mimic-transfected and OGD-induced BMECs detected by Matrigel method; N = 3. The data were expressed as mean ± standard deviation

RT-qPCR results depicted that ODG treatment reduced miR-140-5p expression in BMECs. MiR-140-5p expression was detected in BMECs which had transfected with sh-H19 or oe-H19. It was disclosed that sh-H19 transfection led to an increment of miR-140-5p expression in BMECs while oe-H19 transfection suppressed miR-140-5p expression in BMECs. oe-H19-induced suppression of miR-140-5p expression was rescued by miR-140-5p mimic transfection (Fig. 4E, F).

RETRACTED

In OGD-treated BMECs which were successively transfected with oe-H19 and miR-140-5p mimic, overexpression of miR-140-5p reversed cell viability impairment, increased apoptosis, and decreased migration and angiogenesis caused by H19 upregulation in OGD-treated BMECs (Fig. 4G–J).

### STAT3 Suppression Hinders Apoptosis and Enhances Migration and Angiogenesis of OGD-Induced BMECs

To illustrate the role of STAT3 in OGD-induced BMECs, BMECs were transfected with oe-STAT3 or sh-STAT3. RT-qPCR and Western blot assay examined that sh-STAT3 transfection reduced STAT3 expression while oe-STAT3 transfection elevated STAT3 expression (Fig. 5A, B). STAT3 overexpression ruined cell viability, migration and angiogenesis, and enhanced apoptosis rate. However, STAT3 down-regulation exerted the opposite functions in these parameters in OGD-treated BMECs (Fig. 5C–F).

**Fig. 5:** STAT3 suppression hinders apoptosis and enhances migration and angiogenesis of OGD-induced BMECs. **A** STAT3 mRNA expression in sh-STAT3- or oe-STAT3-transfected and OGD-induced BMECs detected by RT-qPCR; **B** STAT3 protein expression in sh-STAT3- or oe-STAT3-transfected and OGD-induced BMECs detected by western blot assay; **C** Viability of sh-STAT3- or oe-STAT3-transfected and OGD-induced BMECs detected by MTT assay; **D** Cell apoptosis of sh-STAT3- or oe-STAT3-transfected and OGD-induced BMECs detected by flow cytometry; **E** Cell migration of sh-STAT3- or oe-STAT3-transfected and OGD-induced BMECs detected by Transwell assay; **F** Angiogenesis of sh-STAT3- or oe-STAT3-transfected and OGD-induced BMECs detected by Matrigel method; N = 3; *P < 0.05 compared with the oe-NC group; ^#^*P* < 0.05 compared with the sh-NC group. The data were expressed as mean ± standard deviation

RETRACTED

### H19 Binds to miR-140-5p to Modulate STAT3 Expression

The bioinformatics software RNA22 (https://cm.jefferson.edu/rna22/Precomputed/) predicted the binding site of miR-140-5p and STAT3 (Fig. 6A). Dual luciferase reporter gene assay pictured that miR-140-5p inhibited the luciferase activity of the reporter plasmid containing STAT3-WT, suggesting that miR-140-5p binds directly with STAT3 mRNA (Fig. 6B).

**Fig. 6:** H19 binds to miR-140-5p to modulate STAT3. **A** The binding site of miR-140-5p and STAT3 detected by bioinformatics website; **B** The targeted regulatory relationship between miR-140-5p and STAT3 detected by dual luciferase reporter gene assay; **C**–**H** STAT3 expression detected by RT-qPCR and western blot assay; N = 3. The data were expressed as mean ± standard deviation

STAT3 expression in OGD-treated BMECs was detected by RT-qPCR and Western blot assay. It was discovered that up-regulated H19 or down-regulated miR-140-5p increased STAT expression, but H19 inhibition or miR-140-5p overexpression had the opposite effects (Fig. 6C–H). When miR-140-5p and H19 were simultaneously up-regulated, STAT3 expression was retrieved to the basic level. The above results delineated that H19 could regulate STAT3 by binding to miR-140-5p, thereby affecting the viability, migration, apoptosis and angiogenesis of OGD-treated BMECs.

## Discussion

Predominantly topped as the main resource for neonatal death and long-term neurological dysfunction [17], HIBD imposes potent peril on human beings. The co-expression network of lncRNA and miRNA suggests therapeutic potency. Concerning to that, this study mainly elucidated that silencing H19 attenuated HIBD through restoring miR-140-5p and suppressing STAT3.

To begin with, investigations into H19 expression and its functions were conducted and the results delineated that H19 was overexpressed in OGD-treated BMECs, and H19 elimination repressed apoptosis and improved migration and angiogenesis of OGD/R-induced BMECs. At present, the highly expressed H19 is displayed in OGD/R-treated N2a and SH-SY5Y cells in HIE, and H19 up-regulation accelerates cell apoptosis and worsens brain injury [6]. Moreover, an elevation is observed in H19 expression in cerebral I/R injury, and oxidative stress injury is ameliorated which is partially facilitated by depleting H19 [7]. Incremental H19 is exhibited in plasma, white blood cells, and brains of mice with IS [18]. Also, a late study has revealed that H19 is elevated in OGD/R-exposed PC12 cells, and silencing H19 reinforces cell proliferation and impedes cell apoptosis after OGD/R treatment [19]. Additionally, it has been elucidated that H19 is up-regulated in OGD-treated neurons, and transfection of H19 siRNA suppresses apoptosis of OGD-treated neurons in ischemic brain injury [20]. Intriguingly, it is revealed that H19 expression is elevated in OGD-treated cells and its down-regulation protects SH-SY5Y cells from OGD/R-induced cell apoptosis and autophagy in IS [21]. Experimentally, the overexpressed H19 is also found in SH-SY5Y cells treated with OGD/R, and H19 suppression blocks OGD/R-induced cell death in cerebral I/R injury [22].

RETRACTED

Subsequently, the interaction between H19 and miR-140-5p was interpreted in the study. Actually, the precise interplay of H19 and miR-140-5p has not been reported, but the binding relation between H19 and miR-140 has been studied previously [14, 23]. Also, the findings depicted that miR-140-5p was down-regulated in OGD/R-induced BMECs, and its overexpression inhibited apoptosis and promoted migration and angiogenesis of OGD/R-induced BMECs. In fact, miR-140 expression is reduced in HIBD [8]. Currently, a study has illustrated that miR-140-5p up-regulation gives rise to neurological function and hinders cell apoptosis in ICH-induced brain injury [9]. In fact, the action of miR-140-5p in HIBD has been discussed in animal models and the findings demonstrate that miR-140-5p expression is reduced in HIBD rats and miR-140-5p with dexmedetomidine is capable of suppressing cell apoptosis [10]. Whatever, the positive effects of up-regulated miR-140-5p in some brain diseases are in adherence to our study findings.

Moreover, the connection between miR-140-5p and STAT3b was identified. In addition, we found that STAT3 was up-regulated in OGD/R-induced BMECs and its knockdown depressed apoptosis, and attenuated migration and angiogenesis of OGD/R-induced BMECs. Till now, the targeting relation between miR-140-5p and STAT3 has not been convinced yet, which needs further explorations. Exactly, the activated janus kinase (JAK)/STAT3 pathway is manifested in OGD-treated cells, and inhibiting JAK/STAT3 pathway activation ameliorates oxidative stress-induced neuronal injury and enhanced neuronal viability [24]. Besides that, a study has previously demonstrated that disturbance of JAK2/STAT3 signaling reduces neuronal apoptosis which is caused by OGD-activated microglia [25].

## Conclusion

Jointly, the work has proved that H19 bound to miR-140-5p to modulate STAT3 expression, thereby deteriorating HIBD progression. The work has renewed the conception about the pathology and development of HIBD and provided a novel perspective for exploring therapeutic potentials for HIBD patients. Finitely, a large cohort of investigations are required for in-depth comprehension and extension of HIBD management.

RETRACTED

## Supplementary Information

**Additional file 1: Table S1.** Materials. **Table S2.** Primer sequences used in the PCR assay

## Data Availability

The original contributions presented in the study are included in the article/Supplementary Material, further inquiries can be directed to the corresponding author.

## Abbreviations

HIBD: Hypoxic-ischemic brain damage
lncRNA: Long non-coding RAN
STAT3: Signal transducer and activator of transcription 3
BMECs: Brain microvascular endothelial cells
miR: MicroRNA
HIE: Hypoxic ischemia encephalopathy
I/R: Ischemia/reperfusion
IS: Ischemic stroke
ICH: Intracerebral hemorrhage
OGD/R: Oxygen glucose deprivation/reoxygenation
FITC: V-fluorescein isothiocyanate
PI: Propidium iodide
UTR: 3′ Untranslated region
WT: Wild type
MUT: Mutant type
RT-qPCR: Reverse transcription quantitative polymerase chain reaction
GAPDH: Glyceraldehyde-3-phosphate dehydrogenase
RIP: RNA-binding protein immunoprecipitation
ANOVA: Analysis of variance
